The article "Effects of Malaria Parasite Density on Blood Cell Parameters" was published in 2015. Journal: PLoS One.

# Effects of Malaria Parasite Density on Blood Cell Parameters

**DOI:** 10.1371/journal.pone.0121057

**Published:** 2015-03-25

**Authors:** Manas Kotepui, Duangjai Piwkham, Bhukdee PhunPhuech, Nuoil Phiwklam, Chaowanee Chupeerach, Suwit Duangmano

**Affiliations:** 1 Medical Technology Program, School of Allied Health Sciences and Public Health, Walailak University, Nakhon Si Thammarat, Thailand; 2 Medical Technology Laboratory, Phop Phra Hospital, Phop Phra District, Tak Province, Thailand; 3 Institute of Nutrition, Mahidol University, Nakhon Pathom, Thailand; 4 Department of Medical Technology, Faculty of Associated Medical Sciences, Chiang Mai University, Chiang Mai, Thailand; Philipps-University Marburg, GERMANY

## Abstract

Changes in blood cell parameters are already a well-known feature of malarial infections. To add to this information, the objective of this study was to investigate the varying effects that different levels of parasite density have on blood cell parameters. Patients diagnosed with malaria at Phobphra Hospital, Tak Province, Thailand between January 1^st^ 2009 and January 1^st^ 2012 were recruited as subjects for data collection. Blood cell parameters of 2,024 malaria-infected patients were evaluated and statistically analyzed. Neutrophil and platelet counts were significantly higher, however, RBC count was significantly lower in patients with *P*. *falciparum* infection compared to those with *P*. *vivax* infection (p<0.0001). Leukocyte counts were also significantly higher in patients with high parasitemia compared to those with low and moderate parasitemia. In terms of differential leukocyte count, neutrophil count was significantly higher in patients with high parasitemia compared to those with low and moderate parasitemia (p<0.0001). On the other hand, both lymphocyte and monocyte counts were significantly lower in patients with high parasitemia (p<0.0001). RBC count and Hb concentration, as well as platelet count were also significantly reduced (p<0.05) and (p<0.0001), respectively. To summarize, patients infected with different malaria parasites exhibited important distinctive hematological parameters, with neutrophil and eosinophil counts being the two hematological parameters most affected. In addition, patients infected with different malarial densities also exhibited important changes in leukocyte count, platelet count and hemoglobin concentration during the infection. These findings offer the opportunity to recognize and diagnose malaria related anemia, help support the treatment thereof, as well as relieve symptoms of severe malaria in endemic regions.

## Introduction

Changes in blood cell counts are a well-known feature of malarial infections. These changes involve major cell lines including red blood cells (RBC), leukocytes and thrombocytes. Hematological changes in the course of a malaria infection, such as anemia, thrombocytopenia and leukocytosis or leucopoenia are well recognized. These alterations vary with the level of malarial endemicity, background hemoglobinopathy, nutritional status, demographic factors, and also malaria immunity [1,2,3].

Hyperparasitemia has been listed as one of the criterion of severe falciparum malaria by the World Health Organization (WHO) for more than two decades [4]. Previous studies have shown that there is a correlation between parasite density and severity of malarial infections [5,6]. Mortality is also correlated with the degree of parasitemia. Patients with the highest parasite densities also have the highest fatality rates [7]. Additionally, high parasitemia due to *Plasmodium falciparum* infection takes a serious turn in anemia [8]. Moreover, excessive hemolysis of parasitized RBCs in malaria infection may lead to anemia [9]. Thrombocytopenia was also seen in the majority of patients with malaria. It was also observed that at high parasitemias, the platelets were found to be significantly lower. It has been noted by previous studies that increasing levels of *P*. *falciparum* parasite loads results in a decreased platelet count [10,11].

The objective of this study was to demonstrate the impact of *P*. *falciparum* and *P*. *vivax* infections, as well as different parasite densities on blood cell parameters in malaria patients. The hematological parameters (RBC, leukocyte, platelets, hemoglobin level (Hb), mean corpuscular volume (MCV), mean corpuscular hemoglobin (MCH), mean corpuscular hemoglobin concentration (MCHC), and red cell distribution width (RDW) of patients infected with malaria were investigated.

## Methods

### Ethics Statement

This study protocol was reviewed and approved by The Ethical Clearance Committee on Human Rights Related to Researches Involving Human Subjects of Walailak University. The name and Hospital Number (HN) of patients were not revealed. Informed consent was not obtained from research participants, but patient records/information was anonymized and de-identified prior to this analysis.

### Data collection

The data used in this study were collected from the Medical Technology Laboratory Unit, Phobphra Hospital, Tak Province. Data of all patients diagnosed with malaria between January 1st 2009 and January 1st 2012 at Phobphra Hospital, Tak Province, were included in this study. Demographic, clinical and laboratory data of all these patients were collected using a standardized form and information obtained were stored in an electronic database. Leukocyte, red blood cells, and platelet counts were measured using an automatic cell counter. During this study period, three distinct cell counters were independently used after careful calibration (Mindray BC-5180, BC 5300, BC-5200). Absolute numbers of differentiated leukocytes were obtained by the multiplication of the absolute leukocyte counts with their respective differential percentage. Immature or abnormal leukocytes, erythrocytes or platelet clumps were detected, or when cell count results differed substantially from normal values, manual confirmation of automatic cell count results were performed. Other available laboratory examinations included RBC, Hb, MCV, MCH, MCHC, RDW, and platelet counts. The standard procedure used for the diagnosis of malaria is the examination of thick and thin blood smears for malaria parasite by with Wright and Giemsa staining and find organism under light microscopy by laboratorists. After the detection of malarial parasites, thin smears were used to identify the parasite species and parasite density. The level of parasitemia was expressed as percentage (%) of erythrocytes infected with malarial parasites. In this study, one thousand erythrocytes were examined and the numbers of infected-RBC among these were noted. Percent parasitemia was then calculated by dividing the number of infected-RBC by the total number of RBCs indexed and multiplied by 100. The data of patients were divided for comparison into *P*. *falciparum* and *P*. *vivax* groups. For levels of malarial parasitemia, data were grouped into high parasitemia (>10 parasite/ 1 oil field), moderate parasitemia (1–10 parasite/ 1 oil field) and low parasitemia (1–100 parasite/100 oil field) groups. The Kolmogorov-Smirnov test was done. It was found that data were not normally distributed and are therefore presented as medians and range. The demographical parameter, such as gender and nationality, were compared using the Fisher’s Exact Test. Continuous variable, such as age and hematological parameters, were compared using the Mann-Whitney test or Kruskall-Wallis test. Data analysis was performed using SPSS ver. 11.5 (SPSS Inc., Chicago, IL, USA).

## Results

### Patient characteristics

Between January 1^st^ 2009 and December 1^st^ 2012, data from of 2,024 cases of patients with malaria, with all parameters available, were recruited for this study. Of these cases, 987 (48.8%) were caused by *P*. *falciparum*, whereas 1,037 (51.2%) were caused by *P*. *vivax*. No patients with co-infection of *P*. *falciparum* and *P*. *vivax* were found. The median age was significantly different between the 2 groups of parasitic infections (p<0.0001), with significant differences in gender (p = 0.008), nationality (0.012), and also the malarial parasitemia (p<0.0001). There were 1,318 (65.1%) patients with low parasitemia, 542 (26.8%) patients with moderate parasitemia, and 164 (8.1%) patients with high parasitemia. All general characteristics of these patients are shown in Table 1. A consort diagram is also shown in Fig. 1.

**Table 1:** General characteristics.

	***P*.*falciparum* n = 987**	***P*. *vivax***	**P value**	**OR (95%CI)**
		**n = 1,037**		
**Demographic**				
Age	29 (1–92)	26.4 (1–92)	<0.0001*	NA
Male/female, n (%)	626 (63.4%)/361 (36.6%)	598(57.7%)/439(42.3%)	0.008**	1.3 (1.1–1.5)
Thai/Burma/Others, n (%)	460 (46.6%)/496 (50.3%)/31 (3.1%)	549 (52.9%), 465(44.8%), 23 (2.2%)	0.012***	NA
Malarial parasitemia; Low/Moderate/High	527 (53.4%)/309 (31.3%)/151 (15.3%)	791 (76.3%)/233 (22.5%)/13 (1.3%)	<0.0001***	NA

*Comparison of 2 groups using a Mann-Whitney U Test.

**Comparison of 2 groups using Fisher’s Exact Test.

***Comparison of 3 groups using Pearson Chi-Square Test.

**Fig 1:** A consort flow diagram showing the flow of cases through the study.

### Leukocyte, RBC and platelet counts of patients with *P*. *falciparum* and *P*. *vivax* infection

Leukocyte counts were not significantly different in patients with *P*. *falciparum* malaria compared to those with *P*. *vivax* infection (p>0.05) (Table 2). For differential leukocyte counts, neutrophil count was significantly higher in patients with *P*. *falciparum* compared to those with *P*. *vivax* infection (p<0.0001), whereas eosinophil count was lower in patients with *P*. *falciparum* compared to those with *P*. *vivax* infection (p = 0.027). For RBC parameters, RBC count was significantly lower in patients with *P*. *falciparum* compared to those with *P*. *vivax* infection (p = 0.009). In addition, other RBC parameters including MCV, MCH, and MCHC were significantly higher in patients with *P*. *falciparum* compared to those with *P*. *vivax* infection (p<0.05). Platelet count was significantly lower in patients with *P*. *falciparum* compared to those with *P*. *vivax* infection (p<0.0001) (Fig. 2).

**Table 2:** Hematological parameters of different types of malaria infection.

**Parameter**	**Malaria**		**p-value**
	*P*.*falciparum*	*P*.*vivax*	
Leukocyte (x10^3^/μL)	6.47 (5.75)	6.31 (5.69)	0.367
Neutrophil (x10^3^/μL)	67.9 (70)	65.7 (67)	<0.0001*
Lymphocyte (x10^3^/μL)	24.5 (22)	25.7 (23)	0.077
Monocyte (x10^3^/μL)	7 (6)	6.75 (6)	0.061
Eosinophil (x10^3^/μL)	2.74 (2)	3.04 (2)	0.027*
Basophil (x10^3^/μL)	0.93 (1)	0.84 (1)	0.116
RBC (x10^6^/μL)	4.32 (4.39)	4.46 (4.45)	0.009*
Hemoglobin (g/dL)	11.55 (11.9)	11.9 (11.9)	0.21
MCV (fL)	82.5 (83.1)	81 (82)	0.007*
MCH (pg/cell)	27.1 (27.5)	26.6 (27.2)	0.002*
MCHC (g/dL)	33.0 (33.2)	32.8 (33)	0.004*
RDW (%)	13.4 (12.9)	13.4 (13)	0.352
Platelet (x10^3^/μL)	88.4 (73)	97 (84)	<0.0001*

*P-value by Mann-Whitney U Test.

**Fig 2:** Significant differences in the hematological parameters between *P*.*falciparum* and *P*.*vivax* infection.

### Leukocyte, RBC and platelet counts in different parasitemia level

Leukocyte counts were significantly higher in patients with high parasitemia compared to those with low and moderate parasitemia (Table 3). For differential leukocyte counts, neutrophil count was significantly higher in patients with high parasitemia compared to those with low and moderate parasitemia groups (p<0.0001). Both lymphocyte and monocyte count were significantly lower in patients with high parasitemia compared to those with low and moderate parasitemia groups (p<0.0001). RBC count and Hb were significantly reduced in patients with high parasitemia compared to those with low and moderate parasitemia groups (p<0.05), whereas MCV and MCH were significantly reduced in patients with moderate parasitemia compared to those with low and high parasitemia groups (p<0.05). Platelet count was notably reduced in patients with high *parasitemia* compared to those with low and moderate parasitemia groups (p<0.0001) (Fig. 3). It could be predicted that the association between malarial parasitemia and hematological parameters is not influenced by age. Thus, based on the statistical date, age is not a factor that causes any significant differences between malarial parasitemia and hematological variables (Table 4).

**Table 3:** Hematological parameters at different parasitemia levels.

**Parameter**	**Parasitemia level**			**p-value**
	**Low**	**Moderate**	**High**	
Leukocyte (x10^3^/μL)	6.22 (5.6)	6.42 (5.8)	7.63 (6.78)	<0.0001*
Neutrophil (x10^3^/μL)	65.9 (67)	67.2 (70)	72.2 (73)	<0.0001*
Lymphocyte (x10^3^/μL)	25.4 (23)	25.1 (22)	22.9 (21)	0.046*
Monocyte (x10^3^/μL)	7.19 (7)	6.47 (6)	5.57 (5)	<0.0001*
Eosinophil (x10^3^/μL)	2.96 (2)	2.83 (2)	2.52 (2)	0.236
Basophil (x10^3^/μL)	0.88 (1)	0.86 (1)	0.94 (1)	0.431
RBC (x10^6^/μL)	4.41 (4.44)	4.43 (4.45)	4.16 (4.23)	0.001*
Hemoglobin (g/dL)	11.9 (12.1)	11.6 (11.6)	10.9 (10.9)	<0.0001*
MCV (fL)	82.5 (83)	80 (81.1)	81.3 (82.4)	0.001*
MCH (pg/cell)	27 (27.5)	26.5 (26.8)	26.7 (27.1)	0.005*
MCHC (g/dL)	32.9 (33.1)	32.8 (33)	32.9 (33.2)	0.385
RDW (%)	13.3 (12.9)	13.6 (13.1)	13.7 (13)	0.001*
Platelet (x10^3^/μL)	98.9 (84)	85.6 (71)	68.2 (56)	<0.0001*

*P-value by Kruskal Wallis Test.

**Fig 3:** Significant differences in the hematological parameters of various parasite densities of malaria.

**Table 4:** Univariate analysis of malarial parasitemia and hematological parameters adjusted by age of patients.

**Parameters**	**Malarial parasitemia** *	**P value**
Leukocyte (x10^3^/μL)	Moderate	0.268
	High	0.001
Neutrophil (x103/μL)	Moderate	0.042
	High	<0.0001
Lymphocyte (x103/μL)	Moderate	0.646
	High	0.003
Monocyte (x10^3^/μL)	Moderate	<0.0001
	High	<0.0001
RBC (x10^6^/μL)	Moderate	0.493
	High	0.001
Hemoglobin (g/dL)	Moderate	0.105
	High	<0.0001
MCV (fL)	Moderate	<0.0001
	High	0.900
MCH (pg/cell)	Moderate	0.005
	High	0.821
RDW (%)	Moderate	0.001
	High	0.046
Platelet (x10^3^/μL)	Moderate	<0.0001
	High	<0.0001

*The reference category is: Low.

## Discussion

Based on the data collected, infections with *P*. *falciparum* are more serious than infections with other malarial species, particularly *P*. *vivax*, because of the frequency of severe and fatal complications associated with it. This lethal parasite can be the basis to cerebral malaria, acute renal failure, acute malarial hepatitis, hypoglycaemia, hyperpyrexia, non-cardiogenic pulmonary oedema, adult respiratory distress syndrome, adrenal insufficiency-like syndrome, hyperparasitemia, Blackwater fever, cardiac arrhythmias and gastrointestinal syndromes like secretory diarrhea [12,13].

Haematological abnormalities are considered a hallmark of malaria and are reported to be most pronounced in *P*. *falciparum* infections. This study showed that *P*. *falciparum* malaria infections can lead to significant changes of various blood cell parameters compared to infections with *P*. *vivax*, including higher neutrophil and lower eosinophil responses. This finding is found to contrast that of a previous study which reported that malaria induced changes include a reduction in neutrophil levels [14]. The underlying mechanisms include the marginalization of neutrophils to the sites of inflammation, splenic localisation, serum lymphotoxic factors, and intercurrent bacterial infections [15,16,17,18]. Even though the results of this study was found to be different, this study still shows a correlation with another previous study which showed that induced falciparum malaria in Aotus monkeys lead to increase in the absolute neutrophil count post infection [19]. However, leukocytosis was found to be more common in *Plasmodium vivax* infected African American soldiers compared to Caucasian soldiers [20]. For eosinopenia in this study, the previous data showed that *P*. *falciparum* infections can suppress preexisting eosinophilia but *P*. *vivax* infections have less effect on the peripheral blood eosinophil count [21].

This study showed a lower RBC count in *P*. *falciparum* infections compared to than those of *P*. *vivax*. The cause and effect of malaria and anemia is complex and not fully understood. Infected RBCs display a reduced deformability and altered surface characteristics, which usually would lead to them being filtered and cleared by the spleen. However, the malaria parasite *P*. *falciparum* has found a way to counter this protective measure. They modify their host cell membrane, which ultimately results to the cytoadherence of RBCs onto the endothelium. Infected and uninfected erythrocytes cluster together, a process called sequestration and rosetting, and clog up the capillary and postcapillary venules of various organs. In addition, the enhanced destruction of uninfected erythrocytes coupled with a decrease in erythrocyte production all add to malaria related anemia. [22,23]. In accordance with this RBC counts in patients with falciparum malaria was lower than in those patients with vivax malaria. RBC indices including MCV, MCH, and MCHC were also higher in *P*. *falciparum* infection than those of *P*. *vivax* infections. This may be the reason why the rate of RBC production leads to the release of immature RBCs into blood circulation, which may cause an increase in the values of MCV, MCH, and MCHC.

In addition to anemia, a reduction in the number of platelets is another one of the more well-known hematologic changes observed in patients with malaria. This study supported that lower platelet counts among patients infected with *P*. *falciparum* in comparison to those of *P*. *vivax* were notably important. The previous study revealed that the prevalence of thrombocytopenia was similar amongst both infection of vivax and falciparum malaria, but patients with severe falciparum malaria had a significantly lower platelet count compared to the non-severe falciparum malarial patients [24]. Results from other previous studies showed that thrombocytopenia seems to occur through peripheral destruction [25]. Immune-mediated destruction of circulating platelets may be a cause of thrombocytopenia in malaria infections, especially those caused by *P*. *falciparum* [26]. The pathogenic mechanisms by which platelets mediate disease severity in patients with falciparum malaria remains to be delineated. However, clinical studies have shown that platelets in patients with *P*. *falciparum* expressed Toll-like receptors (TLRs), which release prepackaged inflammatory mediators [27] such as Nitric oxide (NO), a key mediator of platelet homeostasis. A decreased bioavailability of NO was found in patients with severe malaria, which may contribute to increased platelet activation and consumption [28,29]. Trends between increasing parasite density and an increase in the level of hematologic parameters were observed in this study. Leukocyte counts, especially neutrophil granulocytes, were significantly higher in patients with high parasitemias compared to those with low and moderate parasitemias. A previous study found a consistent positive relationship between leukocyte counts and parasite density in the Plasmodium-infected patients [30]. Findings of a previous study reported that there was no trend across quartiles of parasite density in relation to leukocyte counts during *P*. *falciparum* and *P*. *vivax* infections [31]. However, lymphocyte and monocyte numbers were significantly higher in patients with low parasitemias compared to those with moderate and high parasitemias. The trend of decreasing platelets with increasing levels of parasitemia observed in this study has been previously noted for *P*. *falciparum* [31,32,33,34] and *P*.*vivax* [31]. Low platelet counts were associated with increased parasite density. This association may result from sensitization induced by parasitized RBCs in platelets, with consequent increase in platelet sensitivity to adenosine diphosphate (ADP) and higher dense-granule secretion [3,35]. These alterations could promote platelet aggregation on the endothelium, such as in cerebral malaria [36].

Anemia can be considered as a measure of the cumulative impact of malaria on an individual patient. Patients with a prolonged history of fever (>2days) were 1.5-fold more likely to anemia and showed a 3-fold reduction in their hematocrit >25% [2]. Although the pathogenesis of anemia in malaria is complex and poorly understood, it is commonly seen in patients with falciparum malaria [8]. It may develop rapidly, taking a serious turn in case of *P*. *falciparum* infection due to a heavy parasite load. At higher levels of parasitemia, excessive hemolysis of parasitized RBCs may lead to anemia. In this study, RBC counts and hemoglobin were significantly reduced in high parasitemia patients, which is consistent with previous studies showing a significant increase in the prevalence of anemia with increase in parasite density [37]. A previous study showed that anemia was observed in 72.4% of patients with a high parasite count, as well as an inverse relationship between parasite densities and hemoglobin levels [38]. The mechanism involving anemia is inconclusive but two possible causes of these alterations are increased hemolysis or a decreased rate of erythrocyte production [39,40]. Moreover, a previous study showed that high parasitemia, even without complications, can lead to high mortality, which can reach up to 50% in patients with parasitemia greater than 10% in areas of low transmission [41]. This information is useful for public health agencies in order to specifically ease malaria related anemia. This should however, be interpreted with caution because it assumes that there are no other factors which are responsible for anemia (confounders).

The main limitation of this study is a confounding factor that may affect hematological parameters such as bacterial, virus, and helminth infections, micronutrient deficiencies, and genetic backgrounds of patients. This study also used microscopy as the only method of detection for malaria parasites; meaning that, some malaria negative patients could have had malarial parasites, which could have been detected by PCR only, and this could have lead to an underestimation of the effect of malarial parasitemia on hematological parameters.

## Conclusion

This study can conclude that patients infected with different malarial parasites exhibit important changes and differences in many hematological parameters with neutrophil and eosinophil count being the two most important changes during malarial infection. In addition, patients infected with different malaria parasite density also exhibit significant in leukocyte count, platelet count and hemoglobin concentration during malarial infection. Policy on malaria control should be pushed towards reducing or clearing malarial parasitic density in the blood.
